This article has been retracted.

# Automatic Detection of Epilepsy Based on Entropy Feature Fusion and Convolutional Neural Network

**DOI:** 10.1155/2022/1322826

**Published:** 2022-05-11

**Authors:** Yongxin Sun, Xiaojuan Chen

**Affiliations:** ^1^College of Electronic Information Engineering, Changchun University of Science and Technology, Changchun, Jilin 130000, China; ^2^College of Physics and Electronic Information, Baicheng Normal University, Baicheng, Jilin 137000, China

## Abstract

Epilepsy is a neurological disorder, caused by various genetic and acquired factors. Electroencephalogram (EEG) is an important means of diagnosis for epilepsy. Aiming at the low efficiency of clinical artificial diagnosis of epilepsy signals, this paper proposes an automatic detection algorithm for epilepsy based on multifeature fusion and convolutional neural network. Firstly, in order to retain the spatial information between multiple adjacent channels, a two-dimensional Eigen matrix is constructed from one-dimensional eigenvectors according to the electrode distribution diagram. According to the feature matrix, sample entropy SE, permutation entropy PE, and fuzzy entropy FE were used for feature extraction. The combined entropy feature is taken as the input information of three-dimensional convolutional neural network, and the automatic detection of epilepsy is realized by convolutional neural network algorithm. Epilepsy detection experiments were performed in CHB-MIT and TUH datasets, respectively. Experimental results show that the performance of the algorithm based on spatial multifeature fusion and convolutional neural network achieves excellent results.

## 1. Introduction

Epilepsy is a common brain disease, and more and more people suffer from it for a long time [1–3]. There are around 65 million people in the world have epilepsy, and the number will reach almost 1 billion by 2030 [4]. The older population aged more than 65 years have higher incidence as one quarter of the new-onsets are diagnosed after this time-point [5]. The individuals with dementias such as Alzheimer's disease have higher risk of developing epilepsy [6–9]. Oxidative stress is an important intrinsic mechanism involved in the development of epilepsy causing brain damage. The imbalance between the antioxidant system and increased oxygen radicals in epilepsy accelerates the process of apoptosis [10]. During seizures, the patient suffers great physical and mental pain. Therefore, automatic detection of epilepsy by techniques such as EEG signals is of great importance.

The seizure of epilepsy has suddenness and repeatability. It causes intense mental pain to patients and their families and reduces their quality of life [11]. When the brain activity of epileptic patients is abnormal, abnormal epileptic discharge often occurs in the EEG signal [12]. The signal includes spike wave, spike slow wave, sharp wave, sharp slow wave, sharp slow complex wave, and sharp slow complex wave. Spikes have sharp waveforms, most of which occur in grand or localized seizures. Spike wave and sharp wave have the same mechanism, longer time than spike wave, reflecting the synchronization degree of discharge. The occurrence of sharp slow complex wave and spinous slow complex wave at different locations or times indicates that there may be multiple abnormal electrical activity regions. At present, the diagnosis of these abnormal signals is still done by doctors through visual observation, based on long-term work experience. This work not only consumes a lot of time and energy of doctors but also has low accuracy. It is difficult for different doctors to reach a common judgment standard, which is highly subjective. Therefore, automatic recognition of epileptic EEG signals can help doctors reduce their workload and assist clinical treatment. It has important practical significance and economic value [13].

In recent years, researches on the recognition of EEG signal mostly reflect the change process of brain transition from one state to another state by extracting the characteristics of time domain, frequency domain [14], time frequency domain [15], linear [16], and nonlinear [17]. The literature [18] shows that in the process of the interaction of multiple brain regions in the brain, the synchronous phenomenon leads to seizures. When a seizure is imminent, seizure-like discharges begin to spread through various pathways in the patient's brain to surrounding brain areas. It then passes through some neural circuits to return to the place where the discharge began, forming a closed circuit. This happens in an endless cycle, transforming the brain's normal, random discharges into a steady, rhythmic discharge. Such an attack mechanism shows that there is a certain correlation between brain regions in the course of the disease. The above characteristics do not fully consider this correlation. Therefore, through the synchronous analysis of the whole brain, it can more truly reflect the changes in the interaction between brain areas during clinical seizures.

With the development of machine learning, more and more intelligent algorithms are applied to EEG signal epilepsy detection. It contains classification methods such as support vector [19], naive Bayes [20], neural network [21], and fuzzy logic system [22]. It also includes principal component analysis (PCA) [23], wavelet packet decomposition (WPD) [24], and the higher order crossings (HOC) [25]. These methods first feature extraction from the original features. Then, a classification model is trained using the new features obtained. Finally, the trained model is used for prediction, so as to achieve the function of epilepsy detection. Although many feature extraction and classification methods have been used in EEG epilepsy detection, it is still an important challenge to extract effective features with rich identification information for subsequent effective detection.

In recent years, as a machine learning method, deep learning has attracted extensive attention in feature learning and other aspects [11]. Deep learning learns the weight of each layer through the desired output. Each layer of the hierarchy adjusts the features to get the features that are more likely to yield the desired output. Each layer optimizes the learning of the input features to obtain more and more discriminating features. In recent years, deep learning technology has been effectively applied in EEG signal processing. Some studies [26–28] have used different feature extraction methods to obtain the characteristics of EEG signals. Then, a convolutional neural network is used to detect epilepsy.

At present, there are only a few literatures that use combined features as the input data of classifier to detect epilepsy. In addition, few literatures have considered the spatial information between electrodes while adopting the combined feature. Therefore, in order to use EEG signals to construct effective features for epilepsy detection, this paper proposes an automatic detection algorithm. The innovations and contributions of this paper are listed below. (1) Single entropy (sample entropy (SE), fuzzy entropy (FE), and permutation entropy (PE)) and different combinations of entropy were input as features to the three-dimensional convolutional neural network for epilepsy detection. (2) Three-dimensional input can not only retain spatial information between electrodes but also integrate various eigenvalues extracted from EEG. The experimental results show that compared with single entropy feature, combined entropy feature can effectively improve the accuracy of epilepsy detection.

The structure of this paper is listed as follows. A related work is described in the next section. The proposed method is expressed in Section 3.  Section 4 focuses on the experiment and analysis.  Section 5 is the conclusion.

## 2. Related Work

### 2.1. Epilepsy Detection

Bioinformatics, medical image processing, and biological signal processing are all applications of intelligent technologies in biomedicine. Bioinformatics studies protein and genetic information. Medical image processing mainly includes analysis of CT and NMR. Biological signal processing is the study of electrical signals such as EEG and ECG. EEG signal is the expression of brain neuron activity and contains a lot of information about human physiological activity. EEG signals have been widely used in the field of epilepsy detection. Epilepsy detection usually involves the use of automated algorithms to analyze a patient's biological signals to determine whether an epileptic is having a seizure or has had one. An important goal of epilepsy detection is to perform this transformation as quickly and efficiently as possible. In recent years, a variety of algorithms for epilepsy detection have been proposed and achieved certain results [13, 14, 29, 30].

There are three kinds of characteristic states of data distribution in EEG signal, which can be roughly distributed as follows: (1) EEG signals of healthy subjects under normal conditions. (2) EEG signals of epileptic patients during the onset, and (3) epileptic intermittent signals. These three signals all contain their own independent data distribution characteristics, and there are certain differences among them [31]. In previous studies, researchers mostly used signal data under state (1) and state (2) with a large amount of known category information to construct classifiers. According to the study, the performance of the classifier will decline if the above classifiers are used to classify and recognize the signal data in state (3), which is different from the data distribution in state (1) and state (2). At the same time, the existing traditional intelligent modeling technology will no longer be applicable. The transfer learning strategies were introduced to cope with the above challenges and achieved satisfactory results.

EEG signals can be divided into the following five categories [12, 31]: (1) EEG signals measured when the healthy volunteers kept their eyes open, (2) EEG signals measured when eyes were closed in healthy subjects, (3) EEG signals of hippocampal structures in patients with epilepsy during interseizure period, (4) EEG signals in epileptic regions of the brain during interseizure period in epileptic patients, and (5) EEG signals measured during seizures in patients with epilepsy, where type (1) and type (2) belong to the signals under state (1). Signals of type (3) and type (4) belong to state (3). Type (5) corresponds to the EEG signal in state (2).

The classifier with transfer learning ability constructed in Reference [15] can classify and recognize signal data in states (1) and (3) with large distribution differences based on EEG signals in states (1) and (2). However, the signals of state (1) in the source domain and target domain EEG signals come from the same subclass. However, when the source domain EEG signals come from type (1) and type (5), and the target domain signals come from type (2) and type (5), the classification recognition effect will be significantly reduced. This is because although both types (1) and (2) are EEG signals measured by healthy people under normal conditions, they still have different distribution characteristics and belong to different classes.

In practical application, the data obtained is incomplete, and the loss of a small type of data often occurs. In this case, simply introducing transfer learning strategy into the classification model construction can not effectively solve this problem. Because these methods only consider the distribution difference between the source domain and the target domain when building the classification model. In feature extraction, the dimension of source and target EEG signals is reduced separately, just like the traditional EEG intelligent recognition method, and the difference of source and target distribution is ignored. Features that contribute greatly to the establishment of classification models in the source domain may not contribute greatly to the recognition of the target domain. However, the features of the source domain which can help the target domain classification and recognition are not selected, which leads to the reduction of the classifier recognition effect.

The recognition of epileptic EEG signal is generally divided into the following steps. Firstly, an appropriate feature extraction method is selected for feature extraction of EEG epileptic signals, and the feature vector set composed of relevant and useful feature information is obtained. Secondly, the training samples are used to model the specific classification methods to get the relevant classifier. Then, the trained classifier is used to classify and recognize other EEG epileptic signals.

### 2.2. Classification and Identification Technology

Since 1990, many intelligent classification methods have been applied to the recognition of EEG signals. The following is a brief description of some common methods.

1. Decision tree algorithm: DT uses induction to generate decision tree and rules in its process and then classifies test data with the obtained decision tree and rules. The decision tree classifier proposed in reference [32] based on fast Fourier transform to extract EEG signal features has achieved better classification accuracy.
2. Naive Bayes algorithm: NB is derived from Bayes' theorem in probability theory, with solid theoretical foundation and high efficiency. The literature [33] proposed a data mining model based on the NB algorithm to realize automatic detection of epilepsy.
3. *K*-nearest neighbor algorithm: KNN helps to determine the class standard of a sample according to the categories of most samples in *K*-nearest neighbors of the sample in its feature space. The KNN classification algorithm based on nonlinear discrete wavelet transform to extract EEG signal features described in literature achieves high classification accuracy.
4. Support vector machine: SVM is considered to be an effective tool to solve the problem of pattern recognition and function estimation [34]. The classification of small samples and high dimensional datasets is particularly effective and has been widely used in EEG intelligent detection.
5. Deep learning algorithm: in recent years, some people have tried to use convolutional neural network to process EEG signals and achieved good results. In the literature [19], the original EEG signals were convolved with convolutional neural network in one dimension to predict epileptic seizures. In [35, 36], the original signal is transformed into the frequency domain through the Fourier transform, and then the convolutional neural network is used for classification.

## 3. The Proposed Method

### 3.1. The Feature of Entropy

#### 3.1.1. Sample Entropy SE

Sample entropy SE represents the rate at which a nonlinear dynamical system generates new modes. The higher the sample entropy, the more complex the sequence. The SE algorithm is as follows:

1. The original sequence phase space *i* = {*i*_1_, *i*_2_, ⋯, *i*_*T*_} is reconstructed to obtain the *w*-dimension vector, as shown follows:

(1) $$\begin{array}{c} I\left(x\right)=\left[i\left(x\right)\;i\left(x+1\right)\cdots i\left(x+w-1\right)\right] \end{array}$$

(2) Calculate the distance between vectors *I*(*x*) and *I*(*y*), and the distance between vectors *I*(*y*) and *I*(*y*) is the one with the largest absolute value of difference between the corresponding elements

(2) $$\begin{array}{c} d\left[I\left(x\right),I\left(y\right)\right]=\max\left\{\left|i\left(x+z\right)-i\left(y+z\right)\right|\right\}, \end{array}$$

where *z* = 1, 2, ⋯, *w* − 1, *x*, *y* = 1, 2, ⋯, *w* − 1

(3) For each *x* value, use *t* to represent the number of *d*[*I*(*x*), *I*(*y*)] less than *r*. Calculate the ratio of this number to the total distance *T* − *w* − 1, and call it *H*_*x*_^*w*^(*r*)

(3) $$\begin{array}{c} H_{x}^{w}\left(r\right)=\frac{t}{T-w-1}. \end{array}$$

The average of all its *x* values is calculated as follows:

(4) $$\begin{array}{c} H^{w}\left(r\right)=\frac{1}{T-w}\overset{T-w}{\underset{x=1}{\sum }}H_{x}^{w}\left(r\right) \end{array}$$

(4) Increase the dimension by 1, and the dimension becomes *w* + 1. Repeat steps (1) to (3) to obtain *H*_*x*_^*w*+1^(*r*), *H*^*w*+1^(*r*)
(5) When the sequence length *t* is finite, the estimated value of sample entropy can be obtained, which can be expressed as

(5) $$\begin{array}{c} \text{SE}=\underset{T⟶\infty }{\lim}\;\left\{-lt\left[\frac{H^{w+1}\left(r\right)}{H^{w}\left(r\right)}\right]\right\} \end{array}$$

#### 3.1.2. Permutation Entropy PE

Permutation entropy PE can measure the randomness of one-dimensional time series. The algorithm has the advantages of simplicity, fast calculation speed, and strong antinoise ability. The basic process is as follows:

1. For sequence *i* = {*i*_1_, *i*_2_, ⋯, *i*_*T*_}  phase space reconstruction, the following equation is obtained:

(6) $$\begin{array}{c} i_{s}\left(n\right)=\left\{i_{s}\left(n\right),i_{s}\left(n+\tau \right),\cdots ,i_{s}\left(n+\left(w-1\right)\tau \right)\right\}, \end{array}$$

where *w* is the embedding dimension and *τ* is the delay time

(2) The reconstructed components in *i*_*s*_(*n*) are arranged in ascending order of numerical size as follows:

(7) $$\begin{array}{c} i_{s}\left[\left(n+\left(y_{1}-1\right)\tau \right)⩽\cdots ⩽\left(n+\left(y_{w}-1\right)\tau \right)\right], \end{array}$$

where *y*_1_, *y*_2_, ⋯, *y*_*w*_ represents the sequence number of each element in the reconstructed sequence, so the sequence number *π* = {*y*_1_, *y*_2_, ⋯, *y*_*w*_} has *w*! different situations

(3) *f*(*π*) is used to represent the frequency of occurrence of each sort mode, then the probability of occurrence of its corresponding sort mode is

(8) $$\begin{array}{c} u_{x}\left(\pi \right)=\frac{f\left(\pi \right)}{\left(T/S\right)-w+1}, \end{array}$$

where 1 ⩽ *x* ⩽ *w*!. According to Shannon entropy definition, the permutation entropy is

(9) $$\begin{array}{c} B_{u}\left(w\right)=-\overset{w!}{\underset{x=1}{\sum }}u_{x}\left(\pi \right)\ln u_{x}\left(\pi \right), \end{array}$$

when *u*_*x*_(*π*) = 1/*w*! and *B*_*u*_(*w*) reaches its maximum ln(*w*!)

(4) Normalize the entropy value, and obtain

(10) $$\begin{array}{c} \text{PE}=\frac{B_{u}\left(w\right)}{\ln\left(w!\right)} \end{array}$$

#### 3.1.3. Fuzzy Entropy FE

Fuzzy entropy (FE) is an improvement of sample entropy SE, which uses exponential function as fuzzy function to measure the similarity of sample entropy. The fuzzy entropy is smoothed by the continuity of exponential function. The specific steps of the algorithm are as follows:

1. Reconstruct the phase space of the original sequence *i* = {*i*_1_, *i*_2_, ⋯, *i*_*T*_} to obtain the *M*-dimension vector, as shown in the following equation:

(11) $$\begin{array}{c} I\left(x\right)=\left[\begin{array}{c} i\left(x\right)\;i\left(x+1\right)\cdots i\left(x+w-1\right) \end{array}\right] \end{array}$$

(2) Calculate the distance between vector *I*(*x*) and *I*(*y*), and the distance between vector *I*(*x*) and *I*(*y*) is the one with the largest absolute value of difference between the corresponding elements, namely,

(12) $$\begin{array}{c} d\left[I\left(x\right),I\left(y\right)\right]=wgi\left\{\left|i\left(x+z\right)-i\left(y+z\right)\right|\right\}, \end{array}$$

where *z* = 1, 2, ⋯, *w* − 1, *x*, *y* = 1, 2, ⋯, *w* − 1

(3) Define the similarity *D*_*xy*_^*w*^ between vector *I*(*x*) and *I*(*y*) by fuzzy function *μ*(*d*_*xy*_^*w*^, *t*, *r*), namely,

(13) $$\begin{array}{c} D_{xy}^{w}=\mu \left(d_{xy}^{w},t,r\right)=e^{-{\left(d_{t}^{w}/r\right)}^{t}}, \end{array}$$

where *t* and *r* are the boundary gradient and width of the fuzzy function, respectively

(4) Define the function as follows:

(14) $$\begin{array}{c} \phi^{w}\left(t,r\right)=\frac{1}{T-w}\overset{T-w}{\underset{x=1}{\sum }}\left(\frac{1}{T-W-1}\overset{T-w}{\underset{y=1,y\neq x}{\sum }}D_{xy}^{w}\right) \end{array}$$

(5) Increase the dimension by 1, and the dimension becomes *w* + 1. Repeat steps (2) to (4) to get *φ*^*w*+1^
(6) The fuzzy entropy is defined as follows:

(15) $$\begin{array}{c} \text{FE}=\ln\phi^{w}\left(t,r\right)-\ln\phi^{w+1}\left(t,r\right) \end{array}$$

### 3.2. Data Preprocessing

The open source datasets CHB-MIT and TUH were used in this experiment. In order to increase the number of samples, the experimental data were segmented. The EEG data for each epileptic seizure and epileptic-free period is of 2 s, and there are 100 instances on average for each class for each patient. In this paper, sample entropy, permutation entropy, and fuzzy entropy are used for feature extraction of EEG signals, respectively. The main method is to extract three kinds of entropy of each EEG channel and get one-dimensional eigenvectors, respectively.

In general, EEG datasets are acquired according to the standard international 10-20 system of electrode distribution of EEG signals.  Figure 1(a) is a plan of the International 10-20 system, where the electrodes used in the actual EEG signal are marked in yellow. In the EEG electrode diagram, you can see that each electrode is adjacent to multiple electrodes. These electrodes record EEG signals in specific areas of the brain. In order to retain the spatial information between multiple adjacent channels, a two-dimensional eigenmatrix (*H* × *W*) was constructed based on the one-dimensional eigenvector according to the electrode distribution diagram in the manner shown in Figure 1, where *H* and *W* of the matrix are the maximum values of the channel in the vertical and horizontal directions, respectively. In this case, both *H* and *W* are equal to 7. In addition, empty channels are filled with zero. In this experiment, three different eigenvalues of EEG signals were extracted from each EEG signal, and the obtained one-dimensional vectors were converted into two-dimensional matrices according to the method shown in Figure 2, and then three two-dimensional matrices were obtained. Then, these three two-dimensional matrices are superimposed into a three-dimensional matrix as the input of CNN. The specific transformation process is shown in Figure 2.

### 3.3. Neural Network Structure

A convolutional neural network is a kind of deep feedforward neural network, which has been widely used in many fields such as image recognition. The CNN has the advantages of good fault tolerance and strong self-learning ability. At the same time, it has the advantages of automatic feature extraction and weight sharing. Through many experiments, the convolutional neural network model is finally constructed by four convolutional layers, a full connection layer, and a softmax layer.

The input of CNN network is a three-dimensional feature matrix composed of two-dimensional feature matrices obtained by three different feature extraction methods. The main function of the pooling layer is to reduce the data dimension. But it comes at the cost of lost information. Due to the small amount of data input from the network in this paper, a pooling layer is not added to the CNN network in this paper in order to retain useful information as much as possible. The specific CNN network model structure is shown in Figure 3. The first convolution layer has 32 feature graphs. The feature graph of the later convolution layer is twice that of the previous one, which is 64, 128, and 256, respectively. The convolution kernel is 3 × 3, and the step is 1. After the convolution operation, SELU activation function is added to make the model have nonlinear feature transformation capability. Then, a full connection layer is connected to map 7 × 7 × 256 feature graphs to feature vector *F* ∈ *R*^1024^. The last part of the network is a softmax classifier, which outputs the result value of epilepsy classification and recognition. In this paper, truncated normal distribution function is used to initialize weights and Adam optimizer is used to minimize cross entropy loss function. The initial learning rate is set to 0.0001. Use Dropout to output with 50% probability to avoid overfitting. In addition, L2 regularization is used to avoid overfitting and improve generalization ability, and the weight of regularization term is set to 0.5.

## 4. Experiment

### 4.1. Experimental Dataset

The hardware devices used in this experiment are Intel I7-11700 CPU and NVIDIA GTX 960 GPU. The experimental software is Python 3.10. At the same time, Google open-source deep learning system TensorFlow is used to build the neural network.

EEG data from Boston Children's Hospital is found in the CHB-MIT dataset [30]. It includes EEG recordings of pediatric patients with refractory epileptic seizures. It collected EEG data from 23 of the 22 subjects. Here, data case CHB21 was obtained from the same female subject 1.5 years after data case CHB01. Each case contains between 9 and 42 consecutives.edf files from a single topic. In most cases, the .edf file contains only one hour of digitized EEG signals. All signals were sampled at a rate of 256 samples per second with 16-bit resolution. Most files contain 23 EEG signals (24 or 26 in some cases). These records were recorded using an international 10-20 EEG electrode location and naming system. In some recordings, other signals were also recorded.

Temple University Hospital (TUH) EEG dataset is the largest EEG dataset available [37]. It included 25,000 EEG recordings and 14,000 cases. It is the total dataset of Temple University Hospital since 2002. EEG signals in this dataset were recorded using Natus Medical Incorporated's Nicolet™ EEG recording technology. The original signal consists of 20 to 128 channel records sampled at the lowest frequency of 250 Hz using a 16-bit A/D converter. Eight types of seizures were recorded, among which focal nonspecific epilepsy, generalized nonspecific epilepsy, and complex partial epilepsy were more common. In the subsequent experiments in this paper, only this three common epilepsy information was detected in the TUH dataset.

### 4.2. Validation of the Algorithm

In this section, the CHB-MIT dataset is used to verify the validity of the algorithm. The experimental results in this section are the results of CHB-MIT dataset sent into the network. Accuracy rate (ACC) and recall rate (REC) are introduced in this paper to measure the performance of classifier comprehensively. Its definition is shown below.

(16) $$\begin{array}{c} \text{ACC}=\frac{\text{TP}+\text{TN}}{\text{TP}+\text{TN}+\text{FN}+\text{FP}}, \end{array}$$

(17) $$\begin{array}{c} \text{REC}=\frac{\text{TP}}{\text{TP}+\text{FN}}, \end{array}$$

where TP and TN are positive and negative samples correctly classified and FP and FN are positive and negative samples incorrectly classified. In this paper, the positive samples are the EEG signals of the “reverse” response, and the negative samples are the EEG signals of the “forward” response.

The selection of feature directly determines the performance of classifier. Classifiers based on different feature combinations have different performance. There are seven input features in this experiment. It includes single entropy feature and combined entropy feature, respectively (SE, PE, FE, SE + PE, SE + FE, PE + FE, and SE + PE + FE). Among them, the sequence of entropy combination has little influence on the recognition accuracy after several comparative experiments. The three-dimensional characteristic matrix is constructed by referring to the above experimental pretreatment methods and steps. SE, PE, and FE are the Eigen matrices of 9 × 9 × 1. SE + PE, SE + FE, and PE + FE are 9 × 9 × 2 eigenmatrices. SE + PE + FE is the Eigen matrix of 9 × 9 × 3. The above 7 Eigen matrices were, respectively, input into the convolutional neural network shown in Figure 3 for experiment. That is, 7 groups of experiments were conducted on each dimension. In addition, this paper also carries on the comparison experiment according to the conventional entropy combination method. In this experiment, the spatial information of EEG electrodes is not considered when constructing the input features; that is, the input features are not converted from one-dimensional feature vector to two-dimensional feature matrix according to the EEG electrode distribution. The seven features without spatial information were input to the one-dimensional convolutional neural network with the same network structure as Figure 3 for experiment, and the experimental Settings were consistent with the neural network Settings proposed in this paper.

In order to verify the influence of single entropy feature, combined entropy feature, and spatial information on epilepsy recognition, this paper conducted experiments on single entropy feature including spatial information, single entropy feature without spatial information, and different combined entropy feature. The results are shown separately in Figure 4. The yellow bar graph in the figure represents the experimental results of the one-dimensional convolutional neural network without spatial information, and the green bar graph represents the experimental results of the neural network proposed in this paper. As can be seen from Figure 4, when comparing the three single entropy features, the classification accuracy of sample entropy as the feature is higher than that of fuzzy entropy and permutation entropy. The accuracy and recall rate of sample entropy in a one-dimensional convolutional neural network are 76.91% and 80.19%, respectively. Compared with single entropy feature, the classification accuracy of combined entropy feature is improved. The average accuracy was the highest when SE + PE + FE was used as the input feature. The average accuracy and recall rate in a one-dimensional convolutional neural network are 86.97% and 87.47%, respectively. The average accuracy and recall rate of the proposed three-dimensional convolutional neural network are 94.36% and 95.57%, respectively, which are 7.39 percentage points and 8.1 percentage points higher than the highest average accuracy of single entropy. Experimental results show that the accuracy of epilepsy detection can be improved significantly when combined entropy is used as the feature input. In addition, the experimental results using spatial information are compared with those using the same type of entropy feature without spatial information. The results show that the detection accuracy of all entropy features using spatial information is higher than that of entropy features without spatial information. When SE + PE + FE was used as the input feature, the average accuracy and recall rate were the highest. Therefore, the experimental results show that the spatial information of EEG electrode distribution can effectively improve the accuracy of epilepsy detection.

In order to further analyze the experimental results of the neural network proposed in this paper, Figures 5(a) and 5(b), respectively, show the accuracy and recall rate of epilepsy detection in different features. As can be seen from the figure, when single entropy is used as the input feature, the accuracy and recall rate of epilepsy detection vary greatly among different subjects. Moreover, its overall accuracy is relatively low. When SE + PE + FE was used as the input feature, the difference of accuracy and recall rate among different subjects was small. And its accuracy rate basically maintains at about 95%. The maximum value of single subject in accuracy and recall rate was 76.91% and 80.19%, respectively. Compared with single entropy as the input feature, when the features of SE + PE + FE was used as the input feature, the classification accuracy of the other subjects improved in both dimensions except for the slight decrease of subject 11 in the arousal dimension. Therefore, the experimental results show that when extracting EEG features, different entropies can be combined to complement each other, thus effectively improving the accuracy of epilepsy detection.

In addition, Figure 6 shows the ROC curve and AUC value of the classification model based on training of different feature combinations. The best value of single entropy is the AUC value of SE, which is only 0.8447. SE + PE + FE had the highest AUC value, which was 0.8837. The feature combination method of the proposed algorithm significantly improves the performance of epilepsy detection.

### 4.3. Comparison of Relevant Algorithms

In order to be further compared with other methods, the algorithms of literature [2], literature [3], literature [13], and literature [24] are selected here for experimental comparison. The TUH dataset is used for comparison experiments. Different from the previous CHB-MIT dataset, the TUH dataset contains three common epilepsy information: focal nonspecific epilepsy, generalized nonspecific epilepsy, and complex partial epilepsy. Therefore, the detection on the TUH dataset is difficult. If we can achieve good performance on this dataset, it will be more beneficial to prove the effectiveness of our proposed method. Finally, the accuracy and recall rate of epilepsy detection are shown in Tables 1 and 2. By observing the results in Tables 1 and 2, the average accuracy and recall rate of the algorithm presented in this paper exceed those of the other four methods.

Meanwhile, by observing the data in Table 2, the highest accuracy and recall rate of the algorithm in this paper are 92.26% and 93.86%. The result in Table 2 is significantly lower than the result in Table 1. This is because there are more types of epilepsy in the TUH dataset, which belongs to multiclassification task. However, in the CHB-MIT dataset, there are only two types of epilepsy and normal data, which belong to the dichotomous task. The multiclassification task is more difficult to detect than the two-classification task, so the performance of the TUH dataset in this paper is lower than that of the CHB-MIT dataset.

## 5. Conclusion

In this paper, the EEG data for each epileptic seizure and epileptic-free period is of 2 s and there are 100 instances on average for each class for each patient, and the entropy value per epoch was calculated, respectively. Transform a one-dimensional vector into a two-dimensional matrix according to the method shown in Figure 1. In this paper, sample entropy, permutation entropy, and fuzzy entropy are analyzed, respectively. Three different eigenvalues of EEG signals were extracted from each EEG signal, and three two-dimensional matrices were obtained. The three two-dimensional matrices and their different combinations were input into the convolutional neural network as features, respectively, for analysis of epilepsy detection in two dimensions of accuracy and recall rate.

The experimental results show that compared with the single entropy feature, the combined entropy feature proposed in this paper can effectively improve the accuracy and recall rate of epilepsy detection. In addition, the spatial information of EEG electrode distribution can effectively improve the accuracy of epilepsy detection. The three-dimensional input convolution neural network combined with the combined entropy feature can retain the spatial information between electrodes and fully extract the EEG signal features. Compared with other relevant methods, the accuracy and recall rate of the proposed method are significantly improved.

## Figures and Tables

**Figure 1:** The transformation of space matrix.

**Figure 2:** The feature extraction process of EEG signal.

**Figure 3:** The structure of proposed neural network.

**Figure 4:** The results of accuracy rate and recall rate in different features.

**Figure 5:** The results of different features.

**Figure 6:** The ROC curves and AUC values in different features.

**Table 1:** The results of CHB-MIT dataset.

Methods	ACC (%)	REC (%)
Literature [2]	82.52	81.67
Literature [3]	86.15	86.59
Literature [13]	88.69	89.76
Literature [24]	91.45	92.24
Proposed	94.36	95.57

**Table 2:** The results of TUH dataset.

Methods	ACC (%)	REC (%)
Literature [2]	80.41	79.56
Literature [3]	84.04	84.48
Literature [13]	86.31	87.42
Literature [24]	89.16	90.33
Proposed	92.26	93.86

## Data Availability

The labeled dataset used to support the findings of this study is available from the corresponding author upon request.
